# Behavioral Training of High-Functioning Autistic Children by Music Education of Occupational Therapy

This article has been retracted.

**DOI:** 10.1155/2022/6040457

**Published:** 2022-09-24

**Authors:** Ting Xia, Zongrun Li

**Affiliations:** Department of Orchestra, Xi'an Conservatory of Music, Xi'an Shaanxi 710061, China

## Abstract

Autistic children, also known as “children from the stars”, have been discovered for more than half a century, but there is still no unified conclusion on the diagnosis, causes, manifestations, and education of autism. The current theory and practice suggest that there is a need to improve the treatment and education of these children. According to existing theories and practices, most autistic children show a special interest in music, and music is very effective in the treatment of autistic children, and through musical activities, children with autism can improve their language, social and emotional, cognitive, and sensorimotor development. In this paper, we record and observe the music classes of children with autism. We select two classes with a total of seven children with autism as the observation subjects in the music classes, record the changes in various aspects and behavioral performance of these seven children with autism in the music activities, and analyze and summarize them. The main purpose of this study is to analyze and summarize how the three major music teaching methods are implemented in the music classroom for autistic children and how they can help autistic children with different characteristics. In the end, we summarize the main problems of music teaching for autistic children found in practice and try to make some suggestions, hoping to provide reference for scholars who study music education for autistic children. The music teaching activities were effective in improving the children's joint attention, movement imitation, rhythm imitation, and cooperation ability, and all three children improved to varying degrees, fulfilling the goals of the teaching activities. The behavioral analysis of the three children during the teaching activities showed that the three children improved their ability to sit comfortably, awareness, musical ability, and rule awareness and reduced inappropriate behaviors and bad emotions, which proved that music education could improve the social and cognitive skills of the children.

## 1. Introduction

The Centers for Disease Control and Prevention released statistics on the prevalence of autism spectrum disorders (ASD), which show that 1 in 54 children is diagnosed with autism [1]. The annual prevalence of autism is on the rise, as in Europe and the United States, and there are currently about 10 million people with autism spectrum disorders, including more than 2 million children under the age of 12 with autism, and the number is increasing year by year [2]. Most special education schools and educational institutions still have problems such as lack of music equipment, insufficient teachers, and limited teachers' teaching skills. In recent years, the state has vigorously advocated “attending classes”, so that children with autism can have the opportunity to receive education together with normal children in ordinary schools, but because some schools do not have special teachers and rehabilitation equipment, they cannot provide rehabilitation training for children with autism in a timely manner [3]. The development of autism education in China is constrained by the lack of special teachers and rehabilitation equipment in some schools, the lack of timely rehabilitation training for autistic children, the attitude of ordinary students towards autistic children, and the failure of children to keep up with the learning progress and the psychological problems of some children [4].

In theory, it is learned that music education involves not only music but also philosophy, aesthetics, psychology, and many other disciplines; in practice, there are not only instrument learning but also many music-related social activities [5]. After a chance encounter with some social activities, it came into contact with “children from the stars” and learned that “children from the stars”, also known as autistic children, are special children [6]. According to the survey, most of the students in special education schools are mainly visually impaired, hearing impaired, and speech impaired, and most of them need parents to accompany them to help them listen to teachers' instructions [7]. The vast majority of children with autism are currently enrolled in schools and receive rehabilitation education, while some children with autism are in special classes in regular kindergartens, or choose to be educated at home [8]. Studies have shown that children with autism have certain deficits in perception, emotion, language, communication, movement, and behavior, and their conditions vary [9]. In this study, we found that although autistic children have certain perceptual deficits, they have certain responses and changes in music and communication with music teachers in the music classroom [10]. Although autistic children refuse to communicate with others through words, music is a pleasant experience for them. Some experiments have shown that most autistic children show a special interest in music and that music therapy is very effective in treating autistic children [11].

The development of autistic children in the areas of language, social and emotional, cognitive skills, and sensorimotor skills is improved through musical activities [12]. During interviews with music teachers and principals in this special education school, we learned that music class is one of their favorite classes. This study will use music pedagogy as the theoretical basis and classroom teaching activities as practice to investigate the use of three major music pedagogies in the classrooms of autistic children, summarize the effects of music therapy models in the field of music education on autistic children in various aspects, and try to propose feasible teaching methods and related suggestions in music education for autism. We also summarize our experiences and make recommendations based on the problems encountered in this music therapy model for researchers related to music education therapy for children with autism. The significance of this paper is that in terms of theory, the cases of music activities are used to increase the practical approach to music therapy in the field of music education and to provide some practical case materials for future researchers in music therapy for children with autism. In terms of practice, cases with different pedagogical theoretical bases are conducted for children with autism with different degrees of symptoms to prove that children with autism have a certain degree of development in language, social and emotional, and cognitive ability. In terms of practice, we have demonstrated that the development of autistic children in the areas of language, social and emotional, cognitive, and perceptual-motor development can be improved and can help autistic children improve their life skills and social adjustment.

In this paper, we record and observe the music classes of children with autism. We select two classes with a total of seven children with autism as observation subjects in the music classes, record the changes in various aspects and behavioral performance of these seven children with autism in the music activities, and analyze and summarize them.

## 2. Related Work

The earliest reference to music therapy in the United States was an unsigned article published in the Columbia Journal in 1789, entitled Music-Physically-Considered, which describes the basic principles of music therapy that have been used to this day and provides evidence of the practice of music therapy in Europe. In the late 1940s, the Music Therapy Society of the National Association of Music Teachers (MTNT) established special programs to educate musicians, physicians, psychiatrists, etc. [13]. In November 1950, the first annual meeting of the National Association for Music Therapy (NAMT) was held jointly with the annual meeting of the National Association of Music Teachers (MTNT) in Washington, DC. In the following years, monthly, quarterly, and annual journals and a number of professional publications were gradually published [14].

The Journal of Music Therapy (JMT) was launched in 1964 and greatly promoted the study of music therapy [15]. To date, the United States has dominated the development of music therapy in the world, and the American Music Therapy Association (AMTA) is also the most authoritative music therapy academic institution in the world. Because research on music therapy began earlier in foreign countries, there are more related research results and monographs [16]. In the conference report of the 30th ISME World Conference, a preconference committee workshop on music in special education, music therapy, and music medicine was recorded. 2012 and 20144 ISME committees on special education music, music therapy, and music medicine were held in Greene and Brazil, respectively [17].

A case study of special education from a federal leadership perspective was published in the Journal of Special Education as part of an illustrative study of federal leadership in special education based on interviews with personnel serving as assistant secretaries and directors of the Office of Special Education Programs in the Special Education and Rehabilitative Services [18]. The research perspective covers the time period from 1967, when the HEW Bureau of Education for Persons with Disabilities was established [19]. A phenomenological approach to interpreting the data reveals that these leaders faced similar barriers in their efforts to implement their vision, that their family background experiences influenced the policies they pursued, that their accomplishments framed the significant evolution of the field, and that their work represents a lifelong commitment to improving education and services for students with disabilities and special needs [20]. It improves and sustains the services needed by people with disabilities [21].

## 3. The Significance of Music Education for the Rehabilitation and Compensation of Autistic Children

### 3.1. Effects of Music Education on Neurological Functions of Children with Autism

Neurologists have proven through numerous experiments that the sound vibrations produced by music have a direct effect on the structure of the human nervous system and the cerebral cortex [22]. When people enjoy music, the music reaches the cerebral cortex through the human senses, and the cerebral cortex can regulate the central nervous system of the human body, convey and act on other nervous systems through the central nervous system, and produce benign regulation and balance on the motor system, cardiovascular system, immune system, and endocrine system, making the children feel happy and tranquil. As autistic children grow up, they gradually realize that they are different from ordinary children, and they may be discriminated against and ridiculed, which may lead to low self-esteem, and these social factors may cause their condition to become more and more serious. Music education can build self-confidence and a sense of success for the child, preparing the individual to adapt to society in the future. Music education can also help parents to reduce the psychological and emotional stress of their children. Most children with autism have severe emotional disturbances. In mild cases, children with autism may laugh and cry for no reason or run and jump for no purpose. We observe the changes in language, social and emotional aspects, cognitive abilities, and sensorimotor aspects of autistic children in the classroom, so as to try to summarize the improvement and impact on autistic children through teaching cases designed by different teaching theories.

Moderate or severe cases are characterized by emotional instability, aggressive behavior (e.g., hitting, biting, and kicking), self-injury (e.g., hitting head and scratching eyes or hair), disturbing others (e.g., screaming and hitting people or objects), and other destructive behaviors. For example, the child must get off at a fixed stop on every bus ride, and getting off one stop early or late can cause a strong emotional response. The child's emotional problems hinder their growth and development and affect their social interactions with others and their mental health. Music education can improve the child's emotional condition and promote the development of social skills. In the process of learning and listening to music, the child's brain can secrete dopamine, which can effectively relieve the child's emotional tension and anxiety, make the child feel relaxed and happy, and reduce the generation of bad emotions. In improvisation, children can express their emotions by hitting the instruments. Relevant studies have shown that after a long period of music education, children's bad emotions and self-injurious behaviors are reduced in frequency, which can make children's emotions become relatively stable and effectively control the generation of bad emotions.

Percussion instruments mainly include percussion blocks, musical bars, triangles, and African drums. During the teaching process, after the child's repeated learning and imitation, it can gradually enhance the child's body coordination, balance and ability to control body muscles, promote the development of the child's gross and fine movements, and greatly help the child to improve intelligence and perceptual ability. Children's songs mainly include many types of songs such as love for the motherland, family, friendship, resource conservation, body parts, plants and animals, fruits, vegetables, festivals, traffic safety education, character education, and general knowledge of life and poems, such as “Family Calling Song”, “Safe Road Song”, and “Fruit Song”. Learning more songs with educational meaning can help improve the abilities of autistic children in various aspects.

Some children with language ability can recite the lyrics completely, which can improve the memory and comprehension ability of the children and improve their cognitive ability to a certain extent. Many studies have shown that music teaching activities can effectively improve children's attention and independent learning ability, and thus promote their cognitive development. Music instruction usually includes articulation exercises, instrument playing, and musical games, which can develop and train autistic children's language skills, imitation skills, cooperation skills, and thus improve their social skills. When children with autism are trained in vocalization and breath training, at the beginning, the child will hum on his or her own. After several imitations, the child gradually changes from a small hum at the beginning to a long sound, which means that sound and breath can be combined together, which is very helpful to promote the development of language skills of children with autism. Vocalization exercises, which focus on vowel sounds, breathing, and vocal tones, can effectively correct the pronunciation problems of children with autism.

### 3.2. A Case Study of Music Education for Children with Autism

The subjects of the study were 3 children with autism, aged between 5 and 7 years old, from the Rehabilitation and Education Center for Special Children. All 3 children were diagnosed with autism by the Linfen Maternal and Child Health Hospital, and rehabilitation training was recommended.  Table 1 shows the basic condition questionnaire and each ability questionnaire of the three children, respectively.

Table 2 combines the rehabilitation training files and VB-MAPP assessments of the three children with autism and shows that the three children have moderate autism, Subject A has a speech disability and Subject B and Subject C have a mental disability, and the cause of the three children's autism is unknown. The three children are currently using rehabilitation training and have no experience with medication.

### 3.3. Language Behavior Milestone Assessment and Placement Plan

The VB-MAPP contains five components, namely Milestone Assessment, Impairment Assessment, Transition Assessment, Task Analysis, and Supportive Competencies. The assessment results provide teachers and parents with a clear picture of the actual developmental age and stage of the child with autism and the abilities achieved and not achieved. The skills assessed by the VB-MAPP scale include requesting, naming, imitative speaking, conversation, listener skills, motor imitation, independent play, social and social play, visual perception and sample matching, language structure, group and classroom skills, and early academics, as shown in Figure 1. The assessment scale is divided into three stages, with a total score of 45 in stage 1, indicating that the child is able to reach a developmental age of 0-18 months. The second stage, with a total score of 60, indicates that the child is able to reach a developmental age of 18-30 months. The total score for stage 3 is 65, indicating that the child is capable of reaching a developmental age of 30-48 months. A score of 1 was assigned when the child was able to perform a task independently, 0.5 if the child was unable to perform it independently and needed the assistance of a bystander, and 0 if the child was unable to perform it even with the demonstration and assistance of a bystander. Rhythmic music and musical instruments can promote the development of physical coordination, such as rhythmic gymnastics, which includes running, spinning, stamping, and clapping.

This assessment scale is a standardized form used by the China Disabled Persons' Federation for the assessment of autistic children. The scale mainly assesses the autistic child's personal situation, basic family information, interests, perception, gross and fine movements, emotions, and behaviors. The file is filled out by the assessor of the designated rehabilitation institution according to the child's rehabilitation training status and assessment results and is kept as an important basis for the child with autism to receive rehabilitation assistance. A “P” in the rehabilitation training file is a “P”, which means that the child completed the training without demonstration or assistance. “E” in the table is not scored, which means that the child failed to complete an item, but had the awareness of the required movement, or could attempt to complete an item after assistance, repeated instructions and demonstration. A score of “F” in the table means that the child cannot complete a certain item. The experimental procedure and data results of this music teaching activity were jointly completed by the author and the evaluator. In order to avoid the subjectivity of the author's behavioral data, the assessor of the rehabilitation center observed and recorded the behavioral data of the three children with autism during the music activity to ensure the objectivity and validity of the experimental results.

## 4. Research Results and Conclusions

### 4.1. Analysis of Rhythm Imitation Results

Figure 2 shows the data of joint attention of three children with autism during the first phase of music activities. The horizontal coordinate indicates the number of sessions of music teaching activities, and the vertical coordinate indicates the percentage of joint attention of the three children. The percentage of joint attention in the first session was 50%. Due to the separation from the parents, Subject A always looked in the direction of the parents during the lesson, and Subject C often got up and ran to his mother or ran to the mirror to sing. The percentage of joint attention in the second session was 57%. Subject A had a better ability to sit still and participated more in the music activity than the other two children. Subject B had a better ability to sit still and pay attention easily, but was also easily attracted to other things. Even though Subject B was able to pay attention, her participation in the classroom tasks was low. Subject C had poor ability to sit comfortably and often ran around the classroom or sang and danced in front of the mirror during the lesson. After the teacher brought him back to his original position several times, it did not take long for Subject C to start running around the classroom again, and his attention was often attracted by other things. In the third lesson, the percentage of joint attention was 73%, which was a great improvement compared to the first two lessons. Subject B started to lie down in class and his jaywalking behavior decreased. Subject C imitated more often and participated in more activities, but sometimes she ran to her parents or played alone, which caused her to lose concentration. By the fourth session, the percentage of joint attention reached 100%, and the goal of this activity was achieved.

Subject B and Subject C showed a decrease in inappropriate behavior and a significant increase in attention and time in the classroom. During the fifth lesson, both Subject B and Subject C's participation in the music activity increased. Subject A's attention was not focused, and Subject A was immersed in his own world for a long time during the lesson, and his participation in the music activity decreased. In the sixth lesson, the percentage of joint attention dropped to 43%. During the lesson, Subject A's attention was still difficult to focus, and he was always distracted and started to stand up or lie down to play. In the seventh session, the percentage of joint attention reached 90%, and Subject A's attention in the class improved significantly, raising the percentage of joint attention. By looking at the results of the data for the seven sessions of joint attention, the goal of the activity was accomplished on one occasion. Compared to the data from the first session, the percentage of joint attention exceeded the first session by 7%-40% on 4 occasions and decreased by about 10% on 1 occasion. The maximum duration of joint attention could reach 6 seconds. The results of the experiment showed that the music teaching activity was effective in improving the joint attention of the 3 children with autism through 7 sessions. The location of this music teaching activity was the rhythm classroom of Linfen Rehabilitation Education Center for Special Children, with an area of 25 square meters, equipped with computers, audio, and electric piano. The musical instruments and equipment needed for this music teaching activity were African drums and sound blocks.

### 4.2. Analysis of Action Imitation Results

Figure 3 shows the movement imitation statistics of three children with autism in the Body Scale Song. The horizontal coordinates indicate the number of sessions of the music activity, and the vertical coordinates indicate the percentage of movement imitation of the three children. Subject A's imitations gradually increased in the first three lessons, then decreased to 27% and 6% in the fifth and sixth lessons, respectively, in which Subject A was unable to concentrate during the lesson, and the percentage of imitations rebounded to 49% in the seventh lesson. Subject B's imitation percentage steadily increased in the seven lessons, although the highest imitation rate only reached 18%, but compared with the first lesson, the number of imitations and the initiative of Subject B were somewhat improved. Subject C shook her head for a long time and could not concentrate during the imitation of movements in the first two lessons, but the highest imitation percentage increased to 90% in the third, fourth, and fifth lessons, and Subject C could actively participate and imitate the teacher's movements in the lessons. Subject B basically did not participate in the “Hello Song” and “Goodbye Song” sessions, but before each session, Subject B sang the complete song in front of the mirror in the classroom and was able to make corresponding movements.

Although Subject A did not achieve the goal of the activity, the highest imitation rate reached 69%, and the imitation rate exceeded 3 times of 22% of the first lesson, which showed a significant improvement of his imitation ability. Subject B also failed to achieve the target of this activity, but the highest imitation rate was 18%, and the imitation rate exceeded 2% of the first session on 5 occasions, so the imitation ability had improved to some extent. Subject C achieved the goal of this activity on one occasion, and the imitation rate exceeded 6% of the first session on three occasions, so there was a significant increase in imitation ability and participation. Thus, it can be seen that this activity is effective in improving the imitation ability of the three autistic children.

## 5. Music Education to Improve the Function of Children with Autism

Children with autism develop a sense of rules and the ability to follow instructions through cooperative tasks that promote the development of social skills. Teaching can be done using sound blocks or xylophones. When choosing songs to work on together, teachers should pay attention to the following: first, choose songs that are familiar, favorite, and simple for the child; second, try to choose songs in major keys. Since most of the children have poor comprehension and lack the sense of rules, in order to reduce the difficulty and avoid frustration of the children, the teacher can grade the tasks and let the students complete them gradually, as shown in Figure 4. First, the teacher first holds the sound block in her hand and the child holds only the mallet in her hand. The teacher holds the sound block in her hand in front of the child and gives instructions for the child to strike it and for the child to cooperate. Second, after several training sessions, the teacher can place a sound block in front of each child, and the child cannot hit the sound block until the teacher gives instructions. Third, after a period of instruction, the teacher can give each child a set of blocks and have the child work together to complete the song. If the child has poor social skills and is grabbing for blocks, then the teacher can leave only one set of blocks and have all children work together to complete the song. The purpose of this is to let the children understand that they can complete their favorite songs through their own efforts and that each child needs to actively participate in order to complete them. This is a great way to develop the child's awareness of the rules and to increase the child's attention span and active participation, thus promoting social skills.

In the sixth lesson, the percentage of imitation dropped to 22%. In the lesson, because Subject A did not actively participate in the activity, she appeared to kneel on the floor or lie down to play, which seriously affected Subject C's learning status and caused her to imitate the movements of Subject A and could not concentrate. In the seventh lesson, the imitation rate of Subject C reached 100%, and the goal of action imitation activity was accomplished.

Subject A's behavior during this stage of music teaching activity was relatively stable, with fewer negative emotions. He was able to remember 2-3 movements in “Hello Song” and was able to imitate some of the lyrics. In the cooperative session of “Tapping the Sound Block”, while the other two children were tapping the sound block, Subject A was able to observe and wait for his turn in the sequence, and this occurred 1-3 times in each session. In the “Passing Game” activity, Subject A was able to follow the rhythm given by the teacher and perform the program. As Subject A only had very little language and did not have the ability to sing, the teacher set the program as “Body Scale Song”. Subject A's ability to remember, imitate speech, and pay attention to the outside world improved, which contributed to his social and cognitive development, as shown in Figure 5. The order of the children's tapping need not be fixed, and the teacher can change the order of tapping in each session, so that the children can learn to understand the instructions and take turns to wait. Once the child understands the instructions and is able to strike the blocks according to the instructions, the teacher can gradually increase the number of blocks for each child.

In the session of “Rhythm Imitation”, Subject B changed from not actively participating at the beginning to actively participating, and her ability to imitate the rhythm improved rapidly. This indicated that the sound block could attract Subject B's attention, stop Subject B's undesirable emotion in time, and reduce Subject B's undesirable emotion and inappropriate behavior. In the “Passing Game” session, when the teacher asked her to perform the program, Subject B took the initiative to sing the upward scales, and since Subject B could not sing the downward scales, the teacher assisted her to do it. Subject B improved his memory of the scales, which contributed to his cognitive development, as shown in Figure 6.

Subject C was able to remember all the movements during the second session of this stage of music teaching, during the “Hello Song” and “Goodbye Song” sessions, and was able to follow the teacher to make the corresponding movements accurately, and when the teacher greeted the other two children, Subject C was able to look at the corresponding children, although this behavior only appeared once, it was already a considerable progress, and to some extent, improved Subject C's social skills. In the fourth session, Subject C was very unstable and the reason for his bad mood was unknown. Subject C then sat down opposite to the teacher and followed the teacher's instruction to hit the sound block, completing the activity of “Hitting the Sound Block”. At this point, the sound block attracted the attention of Subject C and prevented the development of undesirable emotions and inappropriate behaviors. After the fifth session, Subject C no longer grabbed the musical instruments and was able to follow the teacher's instructions to hit them in order, which improved his inability to share objects and promoted his social skills. In the session of “Passing Game”, when it was Subject C's turn to perform a program, Subject C showed strong resistance when the parents reminded him of the name of the program. When the teacher played “Body Scale Song”, Subject C stopped venting his bad emotions and was able to make all the movements accurately following the rhythm of the music without any prompting from the teacher, which was very helpful to the development of his social and cognitive skills. This was helpful for their social and cognitive development. In summary, all three children further improved their imitation and cooperation skills during the second stage of the music activity, and all three children were able to follow the teacher's instructions to complete the tasks in order, improve their behavior of not being able to share objects, reduce the generation of bad emotions, and effectively promote the development of social skills.

## 6. Conclusion

The number of autistic children is increasing year by year, and according to the data, the number of autistic children is increasing at a rate of 10%-18% every year. At present, there are more than one million autistic children, and no complete cure has been found yet, and only different forms of interventions can be used to compensate for their maximum rehabilitation. Through this music teaching activity, the three autistic children improved their social interaction ability to different degrees and showed significant improvement in joint attention, imitation ability, and cooperation ability, in addition, Subject A and Subject B showed concern for others, and Subject B and Subject C had some sense of rules and reduced the number of bad emotions and inappropriate behaviors. It is evident that this music activity was effective in improving the social interaction skills of the three autistic children. The format of this study was music-based, and the author improved the social impairment of three children with autism through two phases of music teaching activities. The children were able to separate from their parents for a short period of time and learn on their own. After 14 sessions of music instruction, the results showed significant improvements in joint attention, imitation, and cooperation in all three children. There were also problems in this study, as the author designed a fragmented teaching content and did not systematically design a music teaching program. Since there were only three children in this study and the duration of the music teaching activities was relatively short, it remains to be verified whether the results of this study and the music teaching methods summarized by the author can have an effect on all children with autism.

## Figures and Tables

**Figure 1:** Verbal behavior milestone assessment.

**Figure 2:** Statistics of common attention results.

**Figure 3:** Action imitation result statistics.

**Figure 4:** Developing a sense of rules for autism improvement.

**Figure 5:** Improved ability to follow instructions in autism.

**Figure 6:** Improved motor imitation in autism.

**Table 1:** Basic information of autistic children.

Basic information	Study Subject A	Study Subject B	Study Subject C
Gender	Male	Female	Male
Age	5 years old	6 years old	5 years old
Diagnosis of autism	Moderate	Moderate	Moderate
VB-MAPP evaluation	75	74	36
Actual developmental age	48 months	45 months	19 months
Whether to take medication	No	No	No

**Table 2:** Questionnaire on various abilities of children with autism.

Capability questionnaire	A	B	C
Imitation ability	Can imitate a single movement or part of a series of body movements	Can imitate part of a single movement or part of a series of body movements	Can imitate a single action or a series of body movements with variation
Social skills	Does not actively call out, can actively participate in some learning activities, can follow most simple instructions, can wait briefly	Does not initiate greetings, talk briefly to strangers, or participate in learning activities. Can follow few, simple instructions	Does not actively greet and interact with peers, does not share toys with others, lacks a sense of discipline, and can follow a few simple instructions
Emotions	Emotional stability, occasional bad moods, less inappropriate behavior	They are emotionally stable and sometimes have bad moods. Inappropriate behaviors such as yelling, crying, etc. occur when their needs are not met	Emotionally unstable, with a high incidence of negative emotions, and when their needs are not met, they may cry loudly, smash things or hurt others
Learning	Sometimes does not actively participate in learning activities and has good patience	Does not actively imitate, does not actively participate in learning activities, has some patience	Strong adaptability, lack of attention and ability to follow directions, often talk to themselves during class, lack of patience, easily absorbed by other objects in the classroom, difficulty concentrating attention
Music preference	I have no obvious interest in music, I seldom listen to songs, I do not know how to sing, and I have never touched any musical instruments.	She likes to listen to children's songs and seldom sings them during the day, but she often plays her children's songs. Never touched any musical instruments	Enjoys listening to upbeat, rhythmic songs, sings a lot, and can sing the words and tones correctly, never touched any musical instrument
Dysfunction	Language skills and social interaction skills	Language skills	Social communication skills

## Data Availability

The data used to support the findings of this study are available from the corresponding author upon request.
